# Effects of Vitamin D on Respiratory Function and Immune Status for Patients with Chronic Obstructive Pulmonary Disease (COPD): A Systematic Review and Meta-Analysis

**DOI:** 10.1155/2022/2910782

**Published:** 2022-03-12

**Authors:** Huan Yang, Deyang Sun, Fengqing Wu, Xiao Xu, Xi Liu, Zhen Wang, Linshui Zhou

**Affiliations:** ^1^The First Clinical College, Zhejiang Chinese Medical University, Hangzhou, Zhejiang 310053, China; ^2^Zhejiang Chinese Medical University, Hangzhou, Zhejiang 310053, China; ^3^The First Affiliated Hospital of Zhejiang Chinese Medical University, Hangzhou, Zhejiang 310006, China

## Abstract

**Background:**

Many studies have demonstrated that vitamin D has clinical benefits when used to treat patients with chronic obstructive pulmonary disease (COPD). However, most of these studies have insufficient samples or inconsistent results. The aim of this meta-analysis was to evaluate the effects of vitamin D therapy in patients with COPD.

**Methods:**

We performed a comprehensive retrieval in the following electronic databases: PubMed, Embase, Cochrane Library, China National Knowledge Infrastructure (CNKI), Wanfang Data, and Chinese Scientific Journals Database (VIP). Two trained reviewers identified relevant studies, extracted data information, and then assessed the methodical quality by the Cochrane risk of bias assessment tool, independently. Then, the meta-analyses were conducted by RevMan 5.4, binary variables were represented by risks ratio (RR), and continuous variables were represented by mean difference (MD) or standardized mean difference (SMD) to assess the efficacy of vitamin D therapy in patients with COPD. Then, publication bias assessment was conducted by funnel plot analysis. Finally, the quality of evidence was assessed by the GRADE system.

**Results:**

A total of 15 articles involving 1598 participants were included in this study. The overall results showed a statistical significance of vitamin D therapy in patients with COPD which can significantly improve forced expiratory volume in 1 second (FEV1) (MD: 5.69, 95% CI: 5.01-6.38,*P* < 0.00001,I2 = 51%) and FEV1/FVC (SMD:0.49, 95% CI: 0.39-0.60,*P* < 0.00001,I2 = 84%); and serum 25 (OH)D (SMD:1.21, 95% CI:1.07-1.34,*P* < 0.00001,I2 = 98%) also increase CD3+ Tcells (MD: 6.67, 95% CI: 5.34-8.00,*P* < 0.00001,I2 = 78%) and CD4+ T cells (MD: 6.00, 95% CI: 5.01-7.00,*P* < 0.00001,I2 = 65%); and T lymphocyte CD4+/CD8+ ratio (MD: 0.41, 95% CI: 0.20-0.61,*P* = 0.0001,I2 = 95%) obviously decrease CD8+ Tcells(SMD: -0.83, 95% CI: -1.05- -0.06,*P* < 0.00001,I2 = 82%), the times of acute exacerbation (RR: 0.40, 95% CI: 0.28-0.59,*P* < 0.00001,I2 = 0%), and COPD assessment test (CAT) score (MD: -3.77, 95% CI: -5.86 - -1.68,*P* = 0.0004,I2 = 79%).

**Conclusions:**

Our analysis indicated that vitamin D used in patients with COPD could improve the lung function (FEV1 and FEV1/FVC), the serum 25(OH)D, CD3+ T cells, CD4 + T cells, and T lymphocyte CD4+/CD8+ ratio and reduce CD8+ T cells, acute exacerbation, and CAT scores.

## 1. Introduction

Chronic obstructive pulmonary disease (COPD) remains one of the most universal chronic lung diseases worldwide, which is a group of chronic airway inflammatory respiratory diseases featured by continuous airflow limitation [1]. As the course of the disease increases, it can lead to airway refactoring [2]. In 2018, the epidemiological study of COPD of China found that the prevalence rate was 14% in people above 40 years old [3]. The World Health Organization (WHO) portends that COPD appears to rank third in death worldwide by 2020, causing a heavy psychological and economic burden on patients [4, 5].

Up to now, the pathological mechanisms of COPD are ascribed to excessive inflammation, dysfunctional oxidative stress, and imbalance of protease-antiprotease. These mechanisms ultimately produce small airway lesions and emphysema lesions, and if two kinds of lesions exist at the same time, the airflow persistence of COPD will be restricted [6]. Smoking as a pathogenic factor, which has an immunosuppressive effect and generally thought to cause respiratory diseases including COPD [6, 7]. However, not all smokers suffer from COPD, and lung inflammation will persist after smoking cessation, so it is speculated that there are autoimmune factors in COPD [8]. When a foreign source of infection invades the body, most COPD patients show immune dysfunction [9], among which T lymphocyte immunity is the main one. T lymphocytes include inhibitory T lymphocytes CD8^+^ and helper T lymphocytes CD4^+^. As a key component, T cell-mediated inflammation can directly destroy lung tissue through T lymphocyte-induced cytotoxicity or indirectly through activating macrophages and eventually cause COPD [10–13]. It has found that the ratio of CD4+/CD8+ T cells in patients with COPD is seriously imbalanced [14]. Besides, CD8^+^T and CD4^+^ T cells as a kind of body immune defense have been verified in the pathogenesis of COPD [15].

Recently, the correlation between vitamin D and COPD has become one of the hot spots in the field of respiratory research [16–18]. In addition to participating in the modulation of bone and calcium-phosphorus metabolism, vitamin D also has an important immunomodulatory effect. 25-hydroxyvitamin D (25(OH)D) is recognized as the optimal indicator of nutritional status of vitamin D [19]. If the body is deficient in vitamin D, it cannot express upregulated antimicrobial peptides, resulting in the persistence of local inflammatory response in lung tissues, damaging lung tissues, and inhibiting emphysema through the homeostasis and function of alveolar macrophages, which is an independent risk of acute exacerbation of COPD (AECOPD) patients [17]. Many clinical studies have demonstrated that vitamin D takes a central part in the prevention and treatment of COPD, which can improve lung function index, lower the frequency of acute attacks, and strengthen St. George's Respiratory Questionnaire (SGRQ) scores and the life quality in COPD patients [20–22]. However, the effect on the T cell immune function in COPD patients still needs further research. Thus, we performed current meta-analysis on the basis of randomized controlled trials (RCTs) to analyze the impact of vitamin D on COPD and to gain evidence-based basis to improve the dysfunctional state of COPD T cells.

## 2. Materials and Methods

### 2.1. Search Procedures

In brief, a program of literature was searched in 6 databases: PubMed, Wanfang database, CQVIP Embase, Cochrane Library, and CNK, from inception to August 2021. Electronic search terms were as follows: “Chronic Obstructive Pulmonary Disease” or “COPD”, as well as “cholecalciferol”, “Vitamin D” or “vit D” or, and “randomized controlled trial” or “RCT”.

### 2.2. Inclusion Criteria

#### 2.2.1. Study Type

RCTs of vitamin D or vitamin D combined with conventional therapy were used as a treatment The researches were available in full in English or Chinese.

#### 2.2.2. Research Object

Diagnosed by imaging or pulmonary function examination; no serious heart, liver, kidney, and other diseases, excluding those with a history of neurological and psychiatric diseases, regardless of race, nationality, or gender, who are diagnosed with stable COPD, the diagnosis is consistent with the “chronic obstructive Guidelines for the diagnosis and therapeutics of lung diseases”.

#### 2.2.3. Intervention Method

The control group received routine treatments (including oxygen therapy, physical exercise, oral theophylline preparations and ambroxol, glucocorticoids, and inhaled long-acting *β*2 receptor agonists), and the experimental group received vitamin D alone or combined intervention with conventional treatments measures of research, and a control study that can verify the therapeutic effect of vitamin D.

#### 2.2.4. Outcome Indicators

Lung function, including FEV1 as well as FEV1/FVC; serum 25(OH)D; subsets of T-lymphocyte, including CD3^+^T/CD4^+^T/CD8^+^T cells, as well as CD4^+^/CD8^+^ratio; acute exacerbation and CAT score.

### 2.3. Exclusion criteria

1. Nonstable patients
2. Noninterventional and non-RCT studies
3. Irrelevant and repeated studies
4. Studies on other lung diseases

### 2.4. Data Extraction and Assessment of Quality

In this section, 2 researchers independently conducted the data extraction based on the inclusion criteria. First author's name, title, publication time, country, age, diagnosis, sample size, intervention measures, treatment time, and outcomes were extracted in each study. The disagreements were resolved by the third researcher. The Cochrane risk of bias tool was detected independently by 2 researchers. The results were appraised as high/low risk or unclear risk. Moreover, the Grading of Recommendations, Assessment, Development, and Evaluation (GRADE) [23] was applied to evaluate the study evidence quality.

### 2.5. Statistical Analysis

Binary variables are represented by risks ratio (RR), and continuous variables are expressed as standardized mean difference (SMD) as well as mean difference (MD), and both are represented by 95% confidence interval (CI). Then, the *χ*^2^ test was used to analyze the statistical heterogeneity. When the statistical results of the heterogeneity *P* ≥ 0.1 and *I*^2^ ≤ 50% among the studies, the fixed effects model (FEM) was employed for the next meta-analysis. In contrast, when the statistical results of heterogeneity *P* ≤ 0.1 and *I*^2^ ≥ 50% among the studies, the random effects model (REM) was adopted for detection. In addition, to ensure the accuracy of the data, a funnel plot was used for publication bias if the number of studies for outcomes was sufficient.

## 3. Results

### 3.1. Searching and Screening Procedure

A total of 798 related studies were enrolled, of which 347 were removed because of duplication. 451 studies were excluded via titles and abstracts because they were incompatible with the inclusion. According to the exclusion criteria, 108 studies were screened out by consulting the full texts; finally, 15 articles [20, 24–37] met our inclusion criteria.  Figure 1 presented the flow chart of the current study.

### 3.2. Characteristics of Studies

17 studies in 15 articles including 1598 patients with samples ranging from 36 to 350.The 17 studies contained 4 methods of administration, oral calcitriol capsules, oral vitamin D, oral liquid calcium, and intramuscular vitamin D. Among these 17 studies, the treatment period ranged from 1 week to 1 year. 15 reports from 13 articles [20, 24–30, 33–37] evaluated the FEV1. 13 studies from 11 articles [20, 24, 25, 27–30, 33, 34, 36, 37] provided data on the FEV1/FVC. 12 trials from 11 articles [20, 24–26, 29–32, 35–37] reported the serum 25(OH) D. 6 trials from 5 articles [28, 30, 31, 34, 36] estimated CD3^+^T cells. 7 studies from 6 articles [28, 30–32, 34, 36] reported the CD4^+^ T cells and CD4^+^/CD8^+^ ratio. 5 studies [28, 30–32, 36] estimated CD8^+^ T cells. 7 studies [20, 24, 26–28, 34, 35] reported the number of acute exacerbations. 4 trials [24, 29, 32, 33] reported the CAT scores. The detailed characteristics of these studies are presented in Table 1.

### 3.3. Quality Assessment

The relative risk of bias in the enrolled studies is presented in Figure 2.

### 3.4. Meta-Analysis

#### 3.4.1. FEV1

A total of 15 studies included were from 13 articles (including 1532 patients: 765 in the study group and 767 in the control). Meta-analysis and heterogeneity test on the impact of vitamin D on FEV1 in patients with COPD indicated that *χ*^2^ = 28.83, *P* = 0.01, *I*^2^ = 51% was heterogeneous, and a REM was employed. The results suggest that the impact of vitamin D supplementation on FEV1 is significant (MD:5.69, 95% CI:5.01-6.38, *P* < 0.0001) (Presented in Figure 3).

#### 3.4.2. FEV1/FVC

13 studies from 11 articles (including 1446 patients: 722 in the study group, 724 in the control group), two groups were compared with FEV1/FVC, the heterogeneity test (*χ*^2^ = 74.58, *P* < 0.00001, *I*^2^ = 84%) with heterogeneity, with REM employed. The results show that in comparison to the control group, vitamin D supplementation can increase the FEV1/FVC of the experimental group and significantly facilitate the lung function of the patients. The difference between the two groups is statistically significant (SMD: 0.49, 95% CI: 0.39-0.60, *P* < 0.00001) (Presented in Figure 4).

#### 3.4.3. Serum 25(OH)D

A total of 12 studies from 11 articles (including 1259 patients: 627 of the study group and 632 of the control) reported the serum 25(OH) D levels of patients. The results of meta-analysis unveiled that the study group was in comparison with the control after supplementation of vitamin D. The heterogeneity test (*χ*^2^ = 454.54, *P* < 0.00001, *I*^2^ = 98%) showed that there was heterogeneity, and the REM was adopted. Serum 25(OH)D combined effect size (SMD:1.21, 95% CI:1.07-1.34, *P* < 0.00001), indicating that serum 25(OH) D in the experimental group was significantly higher than the control (Presented in Figure 5).

#### 3.4.4. CD3^+^T cell

A total of 6 studies from 5 articles (including 609 patients: 306 of the study and 303 of the control). CD3^+^ T cells were compared between the two groups, and the heterogeneity test (*χ*^2^ = 22.43, *P* = 0.0004, *I*^2^ = 78%) with heterogeneity used a random effects model. 6 studies revealed that the number of CD3^+^ T cells in the study group was greater than in the control (MD: 6.67, 95% CI: 5.34-8.00, *P* < 0.00001), indicating that vitamin D supplementation can significantly enhances the percentage of CD3^+^ T cells (Presented in Figure 6).

#### 3.4.5. CD4^+^T cell

7 studies from 6 articles (including 715 patients: 359 of the study and 356 of the control)The CD4^+^ T cell frequency was compared between the two. The heterogeneity test (*χ*^2^ = 17.03, *P* = 0.009, *I*^2^ = 65%) was heterogeneous and used a random effects model. The results suggested that the number of CD4^+^ T cells of the study group was higher than the control (MD: 6.00, 95% CI: 5.01-7.00, *P* < 0.00001). (Presented in Figure 7).

#### 3.4.6. CD8^+^T cell

A total of 5 articles (including 528 patients: 264 of the study, as well as 264 of the control) demonstrated the effect of vitamin D on CD8^+^ T cells. The combined results showed that there was significant heterogeneity between the two (*χ*^2^ = 16.47, *P* = 0.0009, *I*^2^ = 82%), so the REM was employed. 1 study [28] reported that vitamin D treatment did not inhibit CD8^+^ T cells in patients with COPD. In comparison with the control, vitamin D can significantly decline CD8^+^ T cells in patients with COPD (SMD: -0.83, 95% CI: -1.05- -0.61, *P* < 0.00001) (Figure 8).

#### 3.4.7. CD4^+^/CD8^+^ T Cell Ratio

7 studies from 6 articles (including 715 patients: 359 of the study and 356 of the control. The cell ratio of CD4^+^/CD8^+^ T cells was compared between the two groups and there was significantly heterogeneity (*χ*^2^ = 117.71,*P* < 0.00001,*I*^2^ = 95%) , so the REM was employed. In comparison of the control, the vitamin D could significantly improve the cell ratio of CD4^+^/CD8^+^T in patients with COPD (MD: 0.41, 95% CI: 0.20-0.61, *P* = 0.0001) (Figure 9).

#### 3.4.8. Acute Exacerbation

There are 7 studies comparing the number of acute exacerbations in the two groups, and 571 cases (283 patients of the study, as well as 288 patients of the control) were enrolled. The combined results unveiled that there was no heterogeneity between the two (*χ*^2^ = 2.89, *P* = 0.82, *I*^2^ = 0%), so the FEM was employed. The results demonstrated that the frequency of acute exacerbations in the vitamin D group decreased compared to the control (RR: 0.40, 95% CI: 0.28-0.59, *P* < 0.00001), indicating that vitamin D implementation could alleviate the acute exacerbations among patients with COPD. (Figure 10).

#### 3.4.9. CAT Score

A total of 4 studies (involving 289 patients: 145 of the study, as well as 144 of the control) included CAT scores. Overall, due to significant heterogeneity (*χ*^2^ = 14.31, *P* = 0.003, *I*^2^ = 79%), we examined MD via a REM, the results suggested that there were significant differences statistically in terms of CAT (MD: -3.77, 95% CI: -5.86 --1.68, *P* = 0.0004). (Figure 11).

### 3.5. Publication Bias

Perform publication bias analysis on 15 articles, the results show that the inverted funnel chart of FEV1 is basically symmetrical, indicating that there is no obvious publication bias, and the results are more reliable.  Figure 12 presents the funnel plot.

### 3.6. Evidence Quality

In comparing the efficacy of the two groups, the evidence quality is low in the outcome of the FEV1 and FEV1/FVC, CD4^+^, and CD4^+^/CD8^+^.The evidence quality is very low in the four outcomes: the serum 25(OH)D, CD3^+^, CD8^+^,and CAT score, which is owing to the risk of bias, serious inconsistency, indirectness, false, or imprecision. For the outcome of acute exacerbations, the evidence quality is moderate due to the indirectness.  Table 2 presents the summary of findings.

## 4. Discussion

COPD is featured by chronic inflammatory diseases with local and systemic circulation, manifested by small airway lesions and decreased lung tissue elastic function [1]. As the COPD progresses, airway resistance increases, airway structure is remodeled, and collagen fibers increase, causing airway obstruction. Compared with healthy people of the same age, COPD patients often suffer from a decline in immune function, especially in cellular immune function. The percentage of CD3^+^/CD4^+^ T cells of the peripheral blood decreases, while the CD8^+^ T cells increase, and CD4^+^/CD8^+^ ratio is inverted [38]. In addition, there are massive CD8^+^T cells in the small airway wall in the periphery, blood vessel wall, and lung parenchyma in patients with COPD, which makes the ratio of CD8^+^/CD4^+^ increase [38]. Moreover, the percentage of CD8^+^ T cells is positively associated with the emphysema and airflow limitation [39], leading to bacterial colonization on the mucosa of the respiratory tract, causing cough and asthma, so that the disease cannot be better controlled. Studies have revealed that COPD is closely linked to the imbalance of T lymphocyte subsets [40]. T lymphocyte-mediated inflammation is implicated in the occurrence and development of COPD or emphysema [41], as well as CD8^+^T cells within the lungs of patients with COPD. Lymphocytes are directly linked to the airway obstruction [42]. The inheritance and transfer of CD4^+^ lymphocytes after alveolar epithelial cell antigen sensitization led to the occurrence of emphysema in rats, indicating that CD4^+^ lymphocytes may be linked to the pathological process of COPD [43]. Dysfunctional immune responses caused by T lymphocytes play a major role in the occurrence and progression of dysfunctional inflammation of COPD [44]. increasing CD8^+^ T cells remain oneThe lung cytotoxicity of CD8^+^ T cells elevated with the severity of COPD [45]. Studies have shown that the CD8^+^ T cells in the bronchial mucosa (BM) and the severity of airflow obstruction in COPD in stable phase are positively correlated and negatively intertwined with the FEV1% predicted value [46].

As we know, deficiency of Vitamin D is very universal in patients with COPD, and its severity is positively correlated with the degree of serum 25(OH) D deficiency [17]. Vitamin D can affect these inflammatory processes through a variety of mechanisms. Serum 25(OH)D binds to specific vitamin D receptors, acts on lymphocytes, especially T lymphocytes, has immunomodulatory and anti-inflammatory properties, can inhibit their proliferation and differentiation, induce the production of antimicrobial peptides or CD14, and participate respiratory tract inflammation process [47]. An increase in the average level of 25(OH) D can reduce the expression of histocompatibility complex H molecules, leading to the downregulation of costimulatory factors and their release. To inhibit the maturation of dendritic cells [48], it can also induce interleukin-10 to secrete CD4^+^ lymphocytes and regulate T lymphocyte subsets [49]. Studies [50, 51] reported that with the gradual decline of vitamin D levels in patients with COPD, the degree of airway obstruction will gradually increase, and the patients' lung function will also decrease, suggesting that vitamin D levels are important for COPD patients. In this current meta-analysis, vitamin D can facilitate FEV1 and FEV1/FVC and elevate serum 25(OH)D levels. These studies have unveiled that after vitamin D supplementation, the levels of CD3^+^, CD4^+^, and CD4^+^/CD8^+^ in COPD patients increase, and CD8^+^ decrease, which effectively promote the recovery of their cellular immune function, thereby enhancing the patient's immunity as well as their lung function. However, one study showed that CD8^+^ increased, which is intertwined with the heterogeneity, and further research is needed in larger samples. In addition, there are 7 studies showing that vitamin D can reduce the number of AECOPD, and only 4 studies can improve CAT scores. Although only one included study mentioned adverse events, vitamin D supplementation is still an effective therapeutic for most patients with COPD with no serious side effects. Therefore, vitamin D treatment can significantly alleviate COPD. In the prevention and treatment of COPD in the future, proper supplementation of vitamin D is an economical and effective treatment.

However, there is a program of limitations in the present study. First, in this study, a total of 17 RCTs form 15articles were selected, involving 1598 COPD patients. The sample size of the trial was small, and only patients in stable were included. Of note, 3 studies refer to “Global Chronic Obstructive Lung Disease Action (GOLD)” conducted a graded study of patients with A, B, C, and D and did not conduct subgroup analysis. Second, the intervention time of each study, the intervention measures of the control group, and the dosage and administration of vitamin D may also affect the treatment effect. In this study, one study used intramuscular injection, and the rest chose oral administration. We did not conduct a unified analysis on the differences in the use of vitamin D, the dosage, and the therapeutic course. Third, in the 15 enrolled studies, only China has accessed the impact of vitamin D on the T cell subsets of patients with COPD, and the T cells were derived from the COPD patient serum, with no T cell from the sputum or bronchoalveolar lavage fluid in patients with COPD; therefore, further research is needed. Fourth, the current limited evidence shows the use of vitamin D to prevent and treat COPD, and the processing qualities of the enrolled studies are generally low, but these evidences are not enough to recommend vitamin D as a routine program for COPD, and more well-designed and larger scales are needed. The multicenter randomized controlled trial study was further verified, with particular attention to improving the quality of experimental research methodology design.

## 5. Conclusion

The results of this meta-analysis demonstrated that vitamin D can reinvigorate the FEV1, as well as FEV1/FVC within COPD patients, increase serum 25(OH)D, CD3^+^, CD4^+^and CD4^+^/CD8^+^levels, and reduce CD8^+^and the number of acute exacerbations and CAT scores. However, the specific mechanism and the appropriate dose of vitamin D still need to further expand the sample size and extend the follow-up time for further research.

## Figures and Tables

**Figure 1:** Flow chart of the current study.

**Figure 2:** (a) Risk of bias graph. The image shows various possible biases in the meta-analysis. (b) Risk of summary. The image shows various possible risks in the meta-analysis.

**Figure 3:** Forest plot of the FEV1. Meta-analysis and heterogeneity test on the impact of vitamin D on FEV1 in patients with COPD.

**Figure 4:** Forest plot of the FEV1/FVC. The results show that in comparison to the control group, vitamin D supplementation can increase the FEV1/FVC of the experimental group and significantly facilitate the lung function of the patients.

**Figure 5:** Forest plot of the serum 25(OH)D. Meta-analysis unveiled that the study group was in comparison with the control after supplementation of vitamin D.

**Figure 6:** Forest plot of the CD3+ T cells. The results indicate that vitamin D supplementation can significantly enhance the percentage of CD3+ T cells.

**Figure 7:** Forest plot of the CD4+ T cells. The results indicated that the number of CD4+ T cells of the study group was higher than the control.

**Figure 8:** Forest plot of the CD8+ T cells. The results indicate that vitamin D can significantly decline CD8+ T cells in patients with COPD.

**Figure 9:** Forest plot of the CD4+/CD8+ T cells. Vitamin D could significantly improve the cell ratio of CD4+/CD8 + T in patients with COPD.

**Figure 10:** Forest plot of the acute exacerbations. The frequency of acute exacerbations in the vitamin D group decreased compared to the control.

**Figure 11:** Forest plot of the CAT scores. The results indicated that there were significant differences statistically in terms of CAT.

**Figure 12:** Funnel plot of publication bias. The results indicated there is no obvious publication bias.

**(a):** 

Author	Year	Country	Sample size	Cases (T/C)	Age (years)	Diagnosis	Intervention	Couse of treatment	Outcome
An Lehouck	2012	Belgium	150	72/78	T:68 (9) C:68 (8)	Stable COPD	T:100,000 IU monthly of vitamin D, po C: Placebo	1 year	①, ②, ⑦
Ali Alavi Foumani	2019	Iran	63	32/31	T:67.9 ± 7.9 C:68.4 ± 7.8	Stable COPD	T:50,000 IU of vitamin D, po C: Placebo	6 months	①, ②, ⑦, ⑧
Sonja M Bjerk	2013	USA	36	18/18	T:67.6 ± 7 C:68 ± 8	Stable COPD	T:2,000 IU daily of vitamin D, po C: Placebo	6 weeks	①, ②, ⑦
Mojgan Sanjari (calcitriol)	2016	Iran	120	39/42	T:55.6 ± 10.4 C:58.4 ± 9.5	Stable COPD	T: Calcitriol capsules0.25 *μ*g, po, qd, C: Placebo	1 week	①, ②
Mojgan Sanjari (vitamin D)	2016	Iran	120	39/42	T:55.8 ± 9.5 C:58.4 ± 9.5	Stable COPD	T:50,000 IU daily of vitamin D,po C: Placebo	1 week	①, ②
Feng Congrui	2017	China	40	20/20	T:76.73 ± 5.92 C:74.33 ± 6.43	Stable COPD	T:Routinetreatment + calcitriol capsules0.25 *μ*g, po,qd, C: Routine treatment	1 month	①, ⑦
Gu Haiting	2015	China	172	86/86	T:65.95 ± 7.56 C:66.10 ± 7.62	Stable COPD	T:Routine treatment + calcitriol capsules0.25 *μ*g, po,qd C: Routine treatment	6 months	①, ③, ④, ⑤, ⑥, ⑦
Gu Wenchao	2015	China	60	30/30	T:65.37 ± 6.23 C:65.13 ± 7.03	Stable COPD	T:Liquid calcium(1200MG) + vitamin D capsules(1000 IU),po,qd C: Placebo	1 year	①, ②, ⑧
Liu Huige	2018	China	50	25/25	T:64.88 ± 4.62 C:65.62 ± 4.81	Stable COPD	T:Routine treatment + calcitriol capsules0.5 *μ*g/d, po, qd C: Routine treatment	6 months	①, ②, ③, ④, ⑤, ⑥
Ju Junqiang	2015	China	80	40/40	T:68.6 ± 6.2 C:69.4 ± 5.8	Stable COPD	T:Routine treatment + calcitriol capsules0.5 *μ*g/d, po,qd, C: Routine treatment	6 months	②, ③, ④, ⑤, ⑥
Tan Zhixiong	2016	China	106	53/53	T:53.9 ± 7.8 C:54.3 ± 8.6	Stable COPD	T:Routine treatment +3300,000 IU of vitamin D iv, qd C: Routine treatment	2 weeks	②, ③, ⑤, ⑥, ⑧

**(b):** 

Author	Year	Country	Sample size	Cases (T/C)	Age (years)	Diagnosis	Intervention	Couse of treatment	Evaluation index
Wang Qingqing	2019	China	60	30/30	T:70.27 ± 8.30 C:71.37 ± 7.90	Stable COPD	T:Routine treatment +400 IU of vitamin D3, po, bid C: Routine treatment	6 months	①, ⑦, ⑧
Wang Yuehua (A group)	2017	China	141	48/46	T:69.95 ± 3.05 C:67.77 ± 4.34 C:68.4 ± 7.8	Stable COPD	T:Calcitriol capsules0.25 *μ*g/d, po, qd C: Placebo	1 year	①, ③, ⑤, ⑥
Wang Yuehua (B group)	2017	China	141	47/46	T:70.12 ± 1.05 C:67.77 ± 4.34	Stable COPD	T:Calcitriol capsules0.5 *μ*g/d, po, qd C: Placebo	1 year	①, ③, ⑤, ⑥
Wu Shiheng	2020	China	50	25/25	T:64.3 ± 7.94 C:63.6 ± 7.39	Stable COPD	T:Routine treatment +1,600 IU of vitamin D, po, qd C: Routine treatment	6 months	①, ②, ⑦
Zhang Han	2015	China	120	60/60	T:71 ± 10 C:73 ± 9	Stable COPD	T:Routine treatment + calcitriol capsules0.5 *μ*g/d, po, qd C: Routine treatment	6 months	①, ②, ③, ④, ⑤, ⑥
Zhang Tianwei	2014	China	350	175/175	T:66.42 ± 7.20 C:66.38 ± 7.15		T:Routine treatment + calcitriol capsules0.5 *μ*g/d, po, qd C: Routine treatment	3 months	①, ②

①Lung function: (FEV1, FEV1/FVC)①Lung function: (FEV1, FEV1/FVC); ②25(OH)D; ③CD4^+^; ④CD8^+^; ⑤CD4^+^/CD8^+^; ⑥CD3^+^; ⑦Acute Exacerbation; ⑧CAT.

**Table 2:** The summary of findings.

Experimental group vs. control group for COPD							
Patient or population: Patients with COPD Settings: Intervention: Vitamin D or vitamin D + routine treatment Comparison: Placebo or routine treatment							
Outcomes	**Illustrative comparative risks**∗**(95% CI)**			**Relative effect (95% CI)**	**No. of participants (studies)**	**Quality of the evidence (GRADE)**	**Comments**
	Assumed risk	Corresponding risk					
	**Control group**	**Experimental group**					
FEV1		The mean FEV1 in the intervention groups was **5.66 higher** (4.98 to 6.35 higher)			1592 (16 studies)	⊕ ⊕ ⊝⊝ **low**^1^	
FEV1/FVC		The mean FEV1/FVC in the intervention groups was **0.36 standard deviations higher** (0.25 to 0.47 higher)			1336 (12 studies)	⊕ ⊕ ⊝⊝ **low**^1^	SMD 0.36 (0.25 to 0.47)
25(OH)D		The mean 25(OH)D in the intervention groups was **7.32 higher** (7.11 to 7.53 higher)			1259 (12 studies)	⊕⊝⊝⊝ **very low**^1^	
CD3^+^		The mean CD3^+^ in the intervention groups was **6.67 higher** (5.34 to 8 higher)			609 (6 studies)	⊕⊝⊝⊝ **very low**^1^	
CD4^+^		The mean CD4^+^ in the intervention groups was **6 higher** (5.01 to 7 higher)			715 (7 studies)	⊕ ⊕ ⊝⊝ **low**^1^	
CD8^+^		The mean CD8^+^ in the intervention groups was **1.19 lower** (2.4 lower to 0.01 higher)			528 (5 studies)	⊕⊝⊝⊝ **very low**^1^	
CD4^+^/CD8^+^		The mean CD4^+^/CD8^+^ in the intervention groups was **0.41 higher** (0.2 to 0.61 higher)			715 (7 studies)	⊕ ⊕ ⊝⊝ **low**^1^	
Acute exacerbation		**Study population**		**RR 0.4** (0.28 to 0.59)	571 (7 studies)	⊕ ⊕ ⊕⊝ **moderate**^1^	
		**288 per 1000**	**115 per 1000** (81 to 170)				
		**Moderate**					
		**267 per 1000**	**107 per 1000** (75 to 158)				
CAT scores		The mean CAT scores in the intervention groups were **3.77 lower** (5.86 to 1.68 lower)			289 (4 studies)	⊕⊝⊝⊝ **very low**^1^	

^∗^The basis for the **assumed risk** (e.g,. the median control group risk across studies) is provided in footnotes. The **corresponding risk** (and its 95% confidence interval) is based on the assumed risk in the comparison group and the **relative effect** of the intervention (and its 95% CI). **CI:** confidence interval; RR: risk ratio; GRADE: Working Group grades of evidence. **High quality:** Further research is very unlikely to change our confidence in the estimate of effect. **Moderate quality:** Further research is likely to have an important impact on our confidence in the estimate of effect and may change the estimate. **Low quality:** Further research is very likely to have an important impact on our confidence in the estimate of effect and is likely to change the estimate. **Very low quality:** We are very uncertain about the estimate. ^1^ No explanation was provided.

## Data Availability

The datasets used and analyzed during the current study are available from the corresponding author on reasonable request.
